The article "LINC00514 drives osteosarcoma progression through sponging microRNA-708 and consequently increases URGCP expression" was retracted in 2024. Reasons: plagiarized images; overlap with other authors' work; signs of a paper mill; concerns about the images.

# LINC00514 drives osteosarcoma progression through sponging microRNA-708 and consequently increases URGCP expression

**DOI:** 10.18632/aging.103043

**Published:** 2020-04-23

**Authors:** Dapeng Yu, Xiangyan Xu, Sufen Li, Kai Zhang

**Affiliations:** 1 Department of Spine Surgery, Shandong Provincial ENT Hospital, Shandong Provincial ENT Hospital Affiliated to Shandong University, Ji’nan 250022, Shandong, China; 2 Department of Traumatic Orthopedics, Shandong Provincial ENT Hospital, Shandong Provincial ENT Hospital Affiliated to Shandong University, Ji’nan 250022, Shandong, China; 3 Orthopedic and Soft Tissue Surgery, Shandong Cancer Hospital and Institute, Shandong First Medical University and Shandong Academy of Medical Sciences, Ji’nan 250117, Shandong, China; 4 Department of Orthopedics, Shandong Provincial Third Hospital, Ji’nan 250031, Shandong, China

**Keywords:** long noncoding RNA, osteosarcoma, microRNA

## Abstract

Long intergenic nonprotein-coding RNA 00514 (LINC00514) is upregulated in papillary thyroid cancer and contributes to its aggressiveness. In this study, we thoroughly explored the expression profile, specific functions, and relevant molecular mechanism of LINC00514 in osteosarcoma (OS). Herein, LINC00514 was significantly upregulated in OS tissues and cells, and increased LINC00514 expression was closely correlated with tumor size, TNM stage, and distant metastasis. OS patients with high LINC00514 expression had shorter overall survival than those with low LINC00514 expression. LINC00514 interference inhibited OS cell proliferation, colony formation, migration, and invasion *in vitro* but promoted cell apoptosis and G0/G1 cell cycle arrest. LINC00514 downregulation hindered OS tumor growth *in vivo*. Mechanistically, LINC00514 functioned as a competing endogenous RNA by directly interacting with microRNA-708-5p (miR-708) and consequently increasing the expression of upregulator of cell proliferation (URGCP). Both miR-708 knockdown and URGCP restoration partially neutralized anticancer activities of LINC00514 silencing in OS cells. LINC00514 increases URGCP expression by acting as a competing endogenous RNA for miR-708, thus exerting oncogenic roles in OS progression. In conclusion, the LINC00514/miR-708/URGCP pathway may be a promising target for drug discovery in the future.

## INTRODUCTION

Osteosarcoma (OS) is a primary malignant bone tumor originating from mesenchymal cells. Occurring primarily in adolescents and children [1], OS is characteristically destructive and highly metastatic [2]. Its incidence is approximately 4.4 individuals per million globally, and it is mostly distributed in developing and underdeveloped countries [3]. In the past decade, significant developments in diagnostics and therapeutics have notably decreased the mortality rate and improved the clinical outcomes of OS [4]; however, OS remains a serious threat to human health because of its frequent recurrence and distant metastasis [5, 6]. The 5-year survival rate of patients with localized OS is approximately 80%, whereas that of patients diagnosed with metastasis is as low as 15%–30% [7]. Furthermore, approximately 40% patients with advanced OS progress to metastasis during treatment [8]. Complexity of OS pathogenesis is the major obstacle to increasing therapeutic efficacy [9, 10]. Therefore, pivotal mechanisms underlying OS initiation and progression must be revealed to identify novel therapeutic targets and further improve patient prognosis.

The article "LINC00514 drives osteosarcoma progression through sponging microRNA-708 and consequently increases URGCP expression" was retracted in 2024. Reasons: plagiarized images; overlap with other authors' work; signs of a paper mill; concerns about the images.

Long noncoding RNAs (lncRNAs) are >200-nucleotide-long transcripts [11]. LncRNAs are nonprotein-coding RNAs that were considered untranslated and nonfunctional until recently [12]. However, recent studies have demonstrated lncRNA involvement in various physiological and pathological processes [13–15]. LncRNA dysfunction is a key factor in diverse human diseases, particularly cancer [16], with mounting evidence supporting a close association between lncRNAs and human cancers [17–19]. LncRNAs may serve both tumor-promoting and tumor-inhibiting functions during carcinogenesis and cancer progression by modulating gene expression at the epigenetic, transcriptional, post-transcriptional, and post-translational levels [20]. A considerable number of lncRNAs are deregulated in OS, affecting a wide range of associated biological activities [21–23]. Accordingly, in-depth studies of the roles and mechanisms of lncRNAs in OS are critical for developing anticancer treatments.

Long intergenic nonprotein-coding RNA 00514 (LINC00514) is upregulated in papillary thyroid cancer and involved in its aggressiveness [24]; however, the expression profile, specific functions, and relevant molecular mechanisms of LINC00514 in OS have not been thoroughly explored. To this end, we aimed to identify LINC00514 expression profile in OS and determine its clinical significance in OS. In addition, functional experiments were designed to reveal the effects of LINC00514 on the malignant behavior of OS cells *in vitro* and *in vivo*. Precise mechanisms underlying the pro-oncogenic roles of LINC00514 in OS cells were further elucidated through a series of molecular experiments.

## RESULTS

### LINC00514 is upregulated in OS and correlated with poor clinical outcomes

To understand the function of LINC00514 in OS, its expression was first assessed in 59 pairs of OS and adjacent normal tissues by quantitative reverse transcription polymerase chain reaction (RT-qPCR). LINC00514 expression was evidently higher in OS tissues than in adjacent normal tissues (Figure 1A). The 59 patients were divided two groups based on LINC00514 expression using the median LINC00514 expression (exact value: 2.43) in OS patients as the cutoff value (LINC00514-low group, n = 29; LINC00514-high group, n = 30). Notably, high LINC00514 expression was significantly correlated with tumor size (*P* = 0.037), TNM stage (*P* = 0.018), and distant metastasis (*P* = 0.025; Table 1). Moreover, the LINC00514-high group showed a shorter overall survival than the LINC00514-low group (Figure 1B; *P* = 0.035). These data suggested that LINC00514 is strongly associated with OS progression.

The article "LINC00514 drives osteosarcoma progression through sponging microRNA-708 and consequently increases URGCP expression" was retracted in 2024. Reasons: plagiarized images; overlap with other authors' work; signs of a paper mill; concerns about the images.

**Figure 1:** **Long intergenic nonprotein-coding RNA 00514 (LINC00514) is upregulated in osteosarcoma (OS) and indicative of poor clinical outcomes.** (**A**) Quantitative reverse transcription polymerase chain reaction of LINC00514 expression in the 59 pairs of OS and adjacent normal tissue samples. (**B**) Kaplan–Meier survival curves showed that increased LINC00514 expression was associated with reduced overall survival in patients with OS (*P* = 0.035). *P < 0.05.

**Table 1:** Correlation between LINC00514 expression and clinical characteristics of patients with osteosarcoma.

**Clinical characteristic**	**LINC00514**		***P*-value**
	**High expression**	**Low expression**	
Age (years)			0.601
<18	19	16	
≥18	11	13	
Sex			0.435
Male	15	11	
Female	15	18	
Tumor size (cm)			0.037
<5	9	17	
≥5	21	12	
TNM stage			0.018
I or II	12	21	
III or IV	18	8	
Distant metastasis			0.025
Presence	16	24	
Absence	14	5	

*P < 0.05.

### LINC00514 interference suppresses OS cell proliferation, migration, and invasion but promotes cell apoptosis and G0/G1 cell cycle arrest

LINC00514 expression was assessed in the OS cell lines HOS, MG-63, U2OS, and SAOS-2 as well as in the normal human osteoblast cell line hFOB 1.19 using RT-qPCR. LINC00514 was clearly upregulated in all four tested OS cell lines compared with in hFOB 1.19 (Figure 2A). Among the four OS cell lines, HOS and MG-63 showed the highest LINC00514 expression and were thus selected for further experiments.

**Figure 2:** **Effects of long intergenic nonprotein-coding RNA 00514 (LINC00514) knockdown on the proliferation, colony formation, apoptosis, cell cycle, migration, and invasion of osteosarcoma (OS) cells.** (**A**) LINC00514 expression in OS cell lines (HOS, MG-63, U2OS, and SAOS-2) and a normal human osteoblasts cell line (hFOB 1.19) was determined by quantitative reverse transcription polymerase chain reaction (RT-qPCR). (**B**) HOS and MG-63 cells were transfected with si-LINC00514 and si-NC. LINC00514 silencing was verified by RT-qPCR. (**C**) Cell Counting Kit-8 assay was carried out to determine the proliferation of HOS and MG63 cells after LINC00514 was knocked down. (**D**) Colony formation assay presented that the colony-forming ability was impaired in HOS and MG63 cells after LINC00514 knockdown. (**E**, **F**) The apoptosis rate and cell cycle status of HOS and MG63 cells with LINC00514 silencing was tested via flow cytometry analysis. (**G**, **H**) Representative images revealing the transwell migration and invasion assays used to examine the impacts of LINC00514 underexpression on HOS and MG-63 cell migration and invasion. *P < 0.05 and **P < 0.01.

The article "LINC00514 drives osteosarcoma progression through sponging microRNA-708 and consequently increases URGCP expression" was retracted in 2024. Reasons: plagiarized images; overlap with other authors' work; signs of a paper mill; concerns about the images.

To investigate the regulatory roles of LINC00514 in OS oncogenicity, three small interfering RNAs (siRNAs) against LINC00514 expression (si-LINC00514#1, si-LINC00514#2, and si-LINC00514#3) were applied to silence LINC00514, and silencing efficiency was determined by RT-qPCR. RT-qPCR revealed that all three siRNAs reduced LINC00514 expression in HOS and MG-63 cells to varying degrees (Figure 2B). Si-LINC00514#2 exhibited the greatest degree of knockdown and was thus used in further experiments and renamed as si-LINC00514.

Next, Cell Counting Kit-8 (CCK-8) and colony formation assays were performed to examine the effects of LINC00514 on OS cell proliferation. LINC00514 knockdown hindered the proliferation (Figure 2C) and colony formation (Figure 2D) of HOS and MG-63 cells. Additionally, HOS and MG-63 cells with LINC00514 knockdown showed obviously increased apoptosis rates compared with control cells (Figure 2E), as evidenced by flow cytometry. Furthermore, LINC00514 downregulation increased the proportion of cells in the G0/G1 phase but decreased the proportion of cells in the S phase (Figure 2F). Transwell migration and invasion assays were conducted to assess the migratory and invasive abilities of HOS and MG-63 cells after LINC00514 silencing. It was evident that LINC00514-depleted HOS and MG63 cells showed impaired migration (Figure 2G) and invasion (Figure 2H). These results suggested that LINC00514 plays a pro-oncogenic role in OS progression.

### LINC00514 functions as a molecular sponge for microRNA-708-5p (miR-708) in OS cells

Numerous studies have demonstrated that cytoplasmic lncRNAs likely function as competing endogenous RNAs (ceRNAs) to serve as a “sponge/decoy” via miRNA binding and thereby increase miRNA target levels at the post-transcriptional level [25–27]. To understand the role of LINC00514 in promoting OS progression, we determined its subcellular localization in HOS and MG-63 cells. LINC00514 was primarily localized in the cytoplasm of HOS and MG-63 cells (Figure 3A), suggesting that LINC00514 affects OS progression by acting as a ceRNA. Bioinformatics prediction showed that LINC00514 contains a binding site for miR-708 (Figure 3B). Because miR-708 acts as a suppressor of OS progression [28], we further investigated the interaction between LINC00514 and miR-708.

The article "LINC00514 drives osteosarcoma progression through sponging microRNA-708 and consequently increases URGCP expression" was retracted in 2024. Reasons: plagiarized images; overlap with other authors' work; signs of a paper mill; concerns about the images.

**Figure 3:** **Long intergenic nonprotein-coding RNA 00514 (LINC00514) directly interacts with microRNA-708 (miR-708) in OS cells.** (**A**) Distribution of LINC00514 in the cytoplasm and nucleus of HOS and MG-63 cells was analyzed by subcellular fractionation. (**B**) Sequences of the wild-type and mutant miR-708-binding sites in LINC00514. (**C**) Quantitative reverse transcription polymerase chain reaction (RT-qPCR) was performed to assess the efficiency of miR-708 mimic transfection in HOS and MG-63 cells. (**D**) Luciferase reporter assay was performed to demonstrate targeted binding between LINC00514 and miR-708 in HOS and MG-63 cells. (**E**) Relative enrichment of LINC00514 and miR-708 in the coprecipitated RNA was examined by RNA immunoprecipitation assay. (**F**) RT-qPCR was performed to detect miR-708 expression in the 59 pairs of OS and adjacent normal tissue samples. (**G**) Spearman’s correlation analysis illustrated a negative correlation between miR-708 and LINC00514 expressions in the 59 OS tissue samples (r = −0.5731, *P* < 0.0001). (**H**) Relative miR-708 expression was measured by RT-qPCR in HOS and MG-63 cells following transfection with si-LINC00514 or si-NC. *P < 0.05 and **P < 0.01.

Luciferase reporter assay was performed to test whether miR-708 could directly bind to LINC00514. HOS and MG-63 cells were cotransfected with miR-708 mimic or miRNA mimic negative control (miR-NC) and the wild-type (WT)-LINC00514 (contains a WT miR-708-binding site in LINC00514 driving the expression of a luciferase gene) or MUT-LINC006514 (contains a mutant miR-708-binding site in LINC00514) reporter plasmid. First, RT-qPCR confirmed that miR-708 was dramatically upregulated in HOS and MG-63 cells following miR-708 mimic introduction (Figure 3C). Luciferase reporter assay revealed a considerable decrease in luciferase activity of WT-LINC00514 caused by miR-708 overexpression in HOS and MG63 cells; these inhibitory effects of miR-708 upregulation were abrogated in cells transfected with MUT-LINC00514 (Figure 3D). Furthermore, an obvious upregulation of LINC00514 and miR-708 in the anti-AGO2 group was found in HOS and MG63 cells (Figure 3E), further confirming that LINC00514 directly interacted with miR-708 in OS cells.

RT-qPCR of tissue samples revealed lower miR-708 expression in OS tissues than in adjacent normal tissues (Figure 3F). Spearman’s correlation analysis revealed an inverse correlation between miR-708 and LINC00514 expressions in the 59 OS tissue samples (Figure 3G; r = −0.5371, *P* < 0.0001). In addition, LINC00514 downregulation increased miR-708 accumulation in HOS and MG-63 cells compared with in negative control siRNA (si-NC)-transfected cells (Figure 3H). Taken together, these results confirmed that LINC00514 acts as a molecular sponge for miR-708 in OS.

The article "LINC00514 drives osteosarcoma progression through sponging microRNA-708 and consequently increases URGCP expression" was retracted in 2024. Reasons: plagiarized images; overlap with other authors' work; signs of a paper mill; concerns about the images.

### URGCP plays oncogenic roles in OS progression and is positively regulated by LINC00514

Upregulator of cell proliferation (URGCP) is a direct miR-708 target in OS [28]. Nonetheless, to the best of our knowledge, detailed roles of URGCP in OS cells remain unclear at present. Before performing knockout experiments to elucidate the roles of miR-708 in OS cells, HOS and MG-63 cells were transfected with URGCP siRNA (si-URGCP), and the efficiency of URGCP silencing was confirmed through western blotting (Figure 4A). CCK-8 and colony formation assays showed that URGCP downregulation suppressed the proliferation (Figure 4B) and colony formation (Figure 4C) of HOS and MG-63 cells compared with those of si-NC-transfected cells. Moreover, si-URGCP transfection increased apoptosis (Figure 4D) and G0/G1 cell cycle arrest (Figure 4E) in these cells. Furthermore, cell migration (Figure 4F) and invasion (Figure 4G) of HOS and MG-63 cells decreased with URGCP silencing. Thus, URGCP plays an oncogenic role in OS.

**Figure 4:** **URGCP promotes the malignant phenotype of OS cells *in vitro****.* (**A**) Western blotting confirmed URGCP silencing in HOS and MG-63 cells after transfection with si-URGCP. (**B**, **C**) Proliferation and colony formation of URGCP-silenced HOS and MG-63 cells were determined by Cell Counting Kit-8 and colony formation assays, respectively. (**D**, **E**) Flow cytometry analysis was performed to evaluate the effect of URGCP depletion on HOS and MG-63 cell apoptosis and cell cycle distribution. (**F**, **G**) Migrated and invasive URGCP-deficient HOS and MG-63 cells were quantified using transwell migration and invasion assays. *P < 0.05 and **P < 0.01.

Given that LINC00514 is a molecular sponge for miR-708 in OS cells, we investigated whether LINC00514 modulates URGCP expression. HOS and MG-63 cells were transfected with si-LINC00514 or si-NC, and changes in URGCP expression were analyzed by RT-qPCR and western blotting. Decreased LINC00514 expression apparently reduced URGCP expression in HOS and MG-63 cells at the mRNA (Figure 5A) and protein (Figure 5B) levels. To analyze the correlation between LINC00514 and URGCP in OS tissues, we next measured URGCP expression in the 59 pairs of OS and adjacent normal tissues. URGCP was highly expressed in OS tissues (Figure 5C) and positively correlated with LINC00514 expression (Figure 5D; r = 0.6105, *P* < 0.0001). Furthermore, rescue experiments were conducted to determine whether the positive effects of LINC00514 on URGCP expression in OS cells attributed to miR-708 sponging. miR-708 inhibitor (in-miR-708)-transfected HOS and MG-63 cells showed decreased miR-708 expression (Figure 5E), as corroborated by RT-qPCR. LINC00514-depleted HOS and MG-63 cells were further cotransfected with in-miR-708 or miRNA inhibitor negative control (in-miR-NC). After cotransfection, RT-qPCR and western blotting confirmed that the significantly reduced URGCP mRNA (Figure 5F) and protein (Figure 5G) expressions due to LINC00514 depletion were restored by miR-708 inhibition. Thus, LINC00514 acts as a ceRNA for miR-708, thereby increasing URGCP expression in OS cells.

The article "LINC00514 drives osteosarcoma progression through sponging microRNA-708 and consequently increases URGCP expression" was retracted in 2024. Reasons: plagiarized images; overlap with other authors' work; signs of a paper mill; concerns about the images.

**Figure 5:** **Long intergenic nonprotein-coding RNA 00514 (LINC00514) positively regulates URGCP in OS cells by sponging microRNA-708 (miR-708).** (**A**, **B**) Quantitative reverse transcription polymerase chain reaction (RT-qPCR) and western blotting were conducted to measure URGCP mRNA and protein levels, respectively, in LINC00514-depleted HOS and MG-63 cells. (**C**) URGCP mRNA expression in the 59 pairs of OS and adjacent normal tissue samples was determined by RT-qPCR. (**D**) Correlation between LINC00514 and URGCP mRNA expressions in OS tissues was analyzed by Spearman’s correlation analysis (r = 0.6105, *P* < 0.0001). (**E**) Efficiency of in-miR-708 expression transfection in HOS and MG-63 cells was evaluated by RT-qPCR. (**F**, **G**) HOS and MG-63 cells were transfected with si-LINC00514 together with in-miR-708 or in-miR-NC. After transfection, the mRNA and protein levels of URGCP were determined by RT-qPCR and western blotting, respectively. *P < 0.05 and **P < 0.01.

### LINC00514 downregulation inhibits malignant OS phenotypes via the miR-708/URGCP regulatory axis

Rescue experiments were conducted to investigate whether the miR-708/URGCP regulatory axis is implicated in the LINC00514-induced oncogenicity of OS cells. HOS and MG-63 cells were cotransfected with si-LINC00514 and in-miR-708 or in-miR-NC. Proliferation (Figure 6A) and colony formation (Figure 6B) of HOS and MG-63 cells reduced by LINC00514 downregulation were reversed by miR-708 suppression. Flow cytometry revealed that reduced LINC00514 expression increased apoptosis (Figure 6C) and G0/G1 cell cycle arrest (Figure 6D) in HOS and MG-63 cells, which were abolished through in-miR-708 cotransfection. Hindered migratory (Figure 6E) and invasive (Figure 6F) abilities of HOS and MG-63 cells caused by LINC00514 silencing were reversed by miR-708 inhibition.

The article "LINC00514 drives osteosarcoma progression through sponging microRNA-708 and consequently increases URGCP expression" was retracted in 2024. Reasons: plagiarized images; overlap with other authors' work; signs of a paper mill; concerns about the images.

**Figure 6:** **microRNA-708 (miR-708) suppression attenuates the effects of long intergenic nonprotein-coding RNA 00514 (LINC00514) silencing in OS cells.** Si-LINC00514 together with in-miR-708 or in-miR-NC was introduced into HOS and MG-63 cells. The transfected cells were subjected to Cell Counting Kit-8 assay, colony formation assay, flow cytometry, and transwell migration and invasion assays to assess cell proliferation (**A**), colony formation (**B**), apoptosis (**C**), cell cycle (**D**), migration (**E**), and invasion (**F**) *in vitro*. *P < 0.05 and **P < 0.01.

Simultaneously, rescue experiments were performed to determine whether URGCP was essential for the roles of LINC00514 in OS cells. Western blotting confirmed the overexpression efficiency of pc-URGCP (an URGCP overexpression plasmid) in HOS and MG-63 cells (Figure 7A). In HOS and MG-63 cells, LINC00514 interference suppressed proliferation (Figure 7B) and colony formation (Figure 7C, 7D), promoted apoptosis (Figure 7E) and G0/G1 cell cycle arrest (Figure 7F), and attenuated migration (Figure 7G) and invasion (Figure 7H). However, URGCP restoration abrogated these effects of LINC00514 knockdown in HOS and MG-63 cells. These results suggested that LINC00514 exerts its tumorigenic roles by targeting the miR-708/URGCP regulatory axis.

**Figure 7:** **Reintroduction of URGCP reverses the si-long intergenic nonprotein-coding RNA 00514 (LINC00514)-mediated inhibition of the malignant phenotype of OS cells.** (**A**) URGCP protein expression in HOS and MG-63 cells after pc-URGCP or pcDNA3.1 transfection was detected by western blotting. (**B**–**F**) LINC00514-silenced HOS and MG-63 cells were further transfected with pc-URGCP or empty pcDNA3.1 plasmid. Cell proliferation, colony formation, and cell apoptosis and cell cycle status were assessed by Cell Counting Kit-8 assay, colony formation assay, and flow cytometry, respectively. (**G**, **H**) The migratory and invasive abilities of the aforementioned cells were assessed by transwell migration and invasion assays. *P < 0.05 and **P < 0.01.

### Decreased LINC00514 expression impairs OS tumor growth *in vivo*

HOS cells stably transfected with small hairpin RNA (shRNA) targeting LINC00514 (sh-LINC00514) or negative control shRNA (sh-NC) were injected into mice to construct a xenograft model for exploring whether LINC00514 affects OS tumor growth *in vivo*. A representative image of the subcutaneous tumor xenograft taken 1 month after cell inoculation is shown in Figure 8A. Tumor volume was obviously reduced in nude mice injected with HOS cells stably expressing sh-LINC00514 (Figure 8B). Average tumor weight was markedly lower in the sh-LINC00514 group than in the sh-NC group (Figure 8C). Furthermore, RT-qPCR demonstrated that tumor xenografts in the sh-LINC00514 group exhibited significantly lower LINC00514 expression (Figure 8D) and higher miR-708 expression (Figure 8E) than those in the sh-NC group. Moreover, URGCP protein was downregulated in tumor xenografts derived from LINC00514-depleted HOS cells (Figure 8F). Taken together, these results suggested that LINC00514 knockdown impaired OS tumor growth *in vivo* by inhibiting the miR-708/URGCP regulatory axis.

The article "LINC00514 drives osteosarcoma progression through sponging microRNA-708 and consequently increases URGCP expression" was retracted in 2024. Reasons: plagiarized images; overlap with other authors' work; signs of a paper mill; concerns about the images.

**Figure 8:** **Decreased long intergenic nonprotein-coding RNA 00514 (LINC00514) expression attenuates tumor growth of OS cells *in vivo*.** (**A**) Representative image of subcutaneous tumor xenografts collected from the sh-LINC00514 and sh-NC groups. (**B**) Tumor width and length was detected every 4 days for 1 month. Growth curve was plotted using the measurement. (**C**) One month after cell injection, all mice were sacrificed and subcutaneous tumor xenografts were weighed. (**D**, **E**) Quantitative reverse transcription polymerase chain reaction was performed to analyze LINC00514 and microRNA-708 expressions in the excised tumor xenografts. (**F**) URGCP protein level in the excised tumor xenografts was quantified by western blotting. **P < 0.01.

## DISCUSSION

LncRNAs have drawn increasing attention in recent years owing to their roles in tumorigenesis [18, 29, 30]. An increasing number of studies have illustrated that lncRNAs play important roles in OS progression, providing an insight into OS pathogenesis [31–33]. Hence, lncRNAs are potential diagnostic and therapeutic targets for OS. Although numerous lncRNAs are dysregulated in OS, only few lncRNAs have been investigated in detail [34–36]. In this study, LINC00514 expression and its clinical relevance in OS were determined. Moreover, the effects of LINC00514 on OS progression were investigated through a series of experiments. Finally, the relevant molecular mechanism was thoroughly elucidated.

LINC00514 was upregulated in papillary thyroid cancer tissues and cell lines [24]. LINC00514 silencing inhibited the proliferation, migration, and invasion of papillary thyroid cancer cells *in vitro* [24]. Nonetheless, its expression and functions in many other human cancers such as OS remain to be explored. In this study, 59 pairs of OS and adjacent normal tissues were collected and used for determining LINC00514 expression by RT-qPCR. LINC00514 was overexpressed in OS tissues compared with in adjacent normal tissues. To further confirm this observation, LINC00514 expression was detected in a panel of OS cell lines; LINC00514 was highly expressed in all four examined OS cell lines. Elevated LINC00514 expression was closely correlated with tumor size, TNM stage, and distant metastasis. Notably, the overall survival of OS patients with high LINC00514 expression was shorter than that of OS patients with low LINC00514 expression. Functionally, decreased LINC00514 expression suppressed OS cell proliferation, colony formation, migration, and invasion *in vitro*; promoted apoptosis and G0/G1 cell cycle arrest *in vitro*; and hindered tumor growth *in vivo*.

The article "LINC00514 drives osteosarcoma progression through sponging microRNA-708 and consequently increases URGCP expression" was retracted in 2024. Reasons: plagiarized images; overlap with other authors' work; signs of a paper mill; concerns about the images.

Furthermore, mechanisms underlying the pro-oncogenic roles of LINC00514 in OS were demonstrated in detail. The ceRNA hypothesis has been studied extensively, and emerging reports have corroborated the involvement of a complex network of lncRNA/miRNA/mRNA pathways in various human cancers including OS [37]. LncRNAs may function as ceRNAs or miRNA sponges by competitively interacting with miRNA response elements to positively abolish miRNA target suppression [38, 39].

In OS cells, LINC00514 was primarily localized in the cytoplasm, suggesting its role as a ceRNA. Bioinformatics prediction to search for putative miRNAs directly interacting with LINC00514 revealed that miR-708 contained the predicted binding sequence for LINC00514. Direct binding and interaction between LINC00514 and miR-708 in OS cells was further confirmed using dual-luciferase reporter and RNA immunoprecipitation (RIP) assays. Interestingly, miR-708 expression was obviously lower in OS tissues than in adjacent normal tissues, and there was a negative correlation between LINC00514 and miR-708 expression in the 59 OS tissue samples. Furthermore, miR-708 expression was negatively regulated by LINC00514 in OS cells. Moreover, LINC00514 was implicated in the positive regulation of the miR-708 target URGCP, and the effect was demonstrated to be exerted through miR-708 sponging. Collectively, these results suggest that LINC00514 serves as a ceRNA to competitively interact with miR-708, thus decreasing miR-708-induced URGCP suppression.

MiR-708 is involved in various human cancers [40–46] including OS [28]. MiR-708 was downregulated in OS and exerted tumor-suppressing actions by inhibiting cell viability, invasion, and migration but promoting cell apoptosis [28]. Mechanistically, URGCP is the direct target of miR-708 in OS cells [28]. URGCP, also known as upregulated gene 4, expression increased in OS tissues [47], and elevated URGCP expression is reportedly closely associated with OS recurrence and metastasis [47]. Moreover, OS patients with high URGCP expression showed shorter overall and disease-free survival than those with low URGCP expression [47]. However, detailed roles of URGCP deregulation in OS malignancy remain obscure. In this study, a series of functional experiments revealed that URGCP inhibition decreased the proliferation, migration, and invasion but promoted the apoptosis and G0/G1 cell cycle arrest in OS cells. More importantly, miR-708 and URGCP expressions were negatively and positively regulated, respectively, by LINC00514 in OS cells. MiR-708 knockdown or URGCP rescue partially diminished the anticancer effects of LINC00514 silencing on OS cells, suggesting that the miR-708/URGCP axis is pivotal for the tumorigenic roles of LINC00514 in OS. Apparently, the LINC00514/miR-708/URGCP pathway is crucial for OS oncogenesis, indicating that this pathway may serve as a promising target for drug discovery in the future.

The article "LINC00514 drives osteosarcoma progression through sponging microRNA-708 and consequently increases URGCP expression" was retracted in 2024. Reasons: plagiarized images; overlap with other authors' work; signs of a paper mill; concerns about the images.

## CONCLUSIONS

LINC00514 is implicated in the regulatory pathway of OS oncogenicity. LINC00514 increases URGCP expression by acting as a ceRNA for miR-708, thereby exerting oncogenic roles in OS progression. Our findings provide novel insights into OS pathogenesis and propose LINC00514 as an effective diagnostic biomarker, prognostic indicator, and therapeutic target for OS.

## MATERIALS AND METHODS

### Tissue samples and cell lines

OS and adjacent normal tissue samples were collected from 59 patients at Shandong Provincial ENT Hospital. No patient had received preoperative radiotherapy or chemotherapy. Following surgical excision, the collected tissues were immediately frozen and stored in liquid nitrogen for subsequent RNA or protein extraction.

hFOB 1.19 was acquired from the Cell Bank of China Academy of Sciences (Shanghai, China). The cells were cultured in Ham’s F12/Dulbecco’s modified Eagle’s medium (Gibco; Thermo Fisher Scientific, Inc.) at 33.5°C in a humidified 5% CO_2_ atmosphere. HOS and MG-63 (Cell Bank of China Academy of Sciences) were cultured in MEM (Gibco; Thermo Fisher Scientific, Inc.), and U2OS and SAOS-2 (Cell Bank of China Academy of Sciences) were maintained in RPMI-1640 (Gibco; Thermo Fisher Scientific, Inc.) and McCoy’s 5A medium (Sigma-Aldrich, St Louis, MO, USA), respectively. All culture media were supplemented with 10% fetal bovine serum (FBS) and 1% penicillin/streptomycin (all from Gibco; Thermo Fisher Scientific, Inc.). The four OS cell lines were cultured at 37°C in a humidified 5% CO_2_ atmosphere.

### Oligonucleotide and plasmid transfection

Three siRNAs targeting LINC00514 (si-LINC00514#1, si-LINC00514#2, and si-LINC00514#3) were designed to silence endogenous LINC00514. si-URGCP was used to suppress URGCP expression. All these siRNAs and si-NC were designed and chemically synthesized by Guangzhou RiboBio Co., Ltd. (RiboBio, Guangzhou, China). MiR-708 mimic, miR-NC, in-miR-708, and in-miR-NC were purchased from Shanghai GenePharma Co., Ltd. (Shanghai, China). The URGCP overexpression plasmid pCDNA3.1-URGCP (pc-URGCP) and an empty pcDNA3.1 plasmid were obtained from GeneChem Co., Ltd. (Shanghai, China). The OS cells were seeded into 6-well plates 1 day before transfection and transfected with the aforementioned molecular products using Lipofectamine® 2000 (Invitrogen; Thermo Fisher Scientific, Inc., Waltham, MA, USA).

The article "LINC00514 drives osteosarcoma progression through sponging microRNA-708 and consequently increases URGCP expression" was retracted in 2024. Reasons: plagiarized images; overlap with other authors' work; signs of a paper mill; concerns about the images.

### Subcellular fractionation

Nuclear and cytoplasmic fractions of OS cells were separated using Ambion® PARIS™ (Invitrogen; Thermo Fisher Scientific Inc.). Subsequent to subcellular fractionation, RNA in the nuclear and cytoplasmic fractions was extracted and subjected to RT-qPCR. Glyceraldehyde-3-phosphate dehydrogenase (GAPDH) and small nuclear RNA U6 were used as internal controls.

### RT-qPCR

The TRIzol^®^ kit was used to isolate total RNA from tissues and cells. Total RNA was quantified using a NanoDrop spectrophotometer (NanoDrop Technologies; Thermo Fisher Scientific, Inc.). To determine LINC00514 and URGCP mRNA expressions, total RNA was reverse transcribed using the PrimeScript™ RT Reagent Kit (TaKaRa Biotechnology, Co., Ltd., Dalian, China). Next, the generated cDNA was subjected to qPCR using the SYBR Green PCR Master Mix (TaKaRa Biotechnology). LINC00514 and URGCP mRNA expressions were normalized to GAPDH expression. To determine miR-708 expression, the miScript Reverse Transcription Kit (Qiagen GmbH, Hilden, Germany) and miScript SYBR Green PCR Kit (Qiagen GmbH) were used for reverse transcription and qPCR, respectively. U6 served as the endogenous control for miR-708. All reactions were performed on the Applied Biosystems 7500 Real-Time PCR System (Thermo Fisher Scientific, Inc.). Relative gene expression was analyzed using the 2^−ΔΔCt^ method [48].

The primers were designed as follows: LINC00514, 5′- GCTCAACATCTCACTTCTCCCAC-3′ (forward) and 5′- CCTTCAGTGTCTGGGAAAGAGAG-3′ (reverse); miR-708, 5′-GGCGCGCAAGGAGCTTACAATC-3′ (forward) and 5′-GTGCAGGGTCCGAGGTAT-3′ (reverse); URGCP, 5′-CTTCATCCTGAGTCCCTACCG-3′ (forward) and 5′-GCCGTTCTGCTGCATTCG-3′ (reverse); U6, 5′-GCTTCGGCAGCACATATACTAAAAT-3′ (forward) and 5′-CGCTTCACGAATTTGCGTGTCAT-3′ (reverse); and GAPDH, 5′-CGGAGTCAACGGATTTGGTCGTAT-3′ (forward) and 5′-AGCCTTCTCCATGGTGGTGAAGAC-3′ (reverse).

### CCK-8 assay

Transfected cells were detached using 0.05% trypsin–EDTA (Gibco; Thermo Fisher Scientific, Inc.) after 24 h of culture, centrifuged, and resuspended in the culture medium. Cell suspension was adjusted to a concentration of 2 × 10^4^ cells/mL and added (100 μL) to each well of a 96-well plate. After 0, 24, 48, and 72 h of culture, cell proliferation was assessed by incubation with 10 μL CCK-8 reagent (Dojindo, Kumamoto, Japan) at 37°C in a humidified 5% CO_2_ atmosphere for an additional 2 h. Absorbance at a wavelength of 450 nm was detected using a microplate reader (Bio-Rad, Hercules, CA, USA).

The article "LINC00514 drives osteosarcoma progression through sponging microRNA-708 and consequently increases URGCP expression" was retracted in 2024. Reasons: plagiarized images; overlap with other authors' work; signs of a paper mill; concerns about the images.

### Colony formation assay

Transfected cells were harvested 24 h after transfection, centrifuged, seeded into 6-well plates at a density of 1 ×10^3^ cells/well, and cultured at 37°C in a humidified 5% CO_2_ atmosphere for 2 weeks. After extensive washing with phosphate-buffered saline, the cells were fixed in 4% paraformaldehyde at room temperature for 20 min and stained with 0.5% crystal violet at room temperature for 20 min. The colonies were observed and counted under an inverted microscope (Olympus Corporation, Tokyo, Japan).

### Flow cytometry

Cell apoptosis was assessed using the Annexin V-FITC Apoptosis Detection Kit (Biolegend, San Diego, CA, USA). Briefly, transfected cells were cultured at 37°C for 48 h, collected using EDTA-free trypsin, and washed with precooled phosphate-buffered saline. After centrifugation at 4°C, cells were resuspended in 100 μL binding buffer and subjected to double staining with 5 μL FITC–Annexin V for 15 min and 10 μL propidium iodide (PI) for 15 min in the dark. Apoptotic cells were detected by flow cytometry (FACScan; BD Biosciences, Franklin Lakes, NJ, USA).

Transfected cells were collected and washed as described above. After fixing overnight in 70% ethanol at 4°C, the transfected cells were collected by centrifugation and treated with 50 μL RNase (100 μg/mL) at 37°C for 20 min. Subsequently, the cells were incubated at room temperature with 500 μL cell-staining buffer supplemented with 25 μL PI (Biolegend). Cells in the G0/G1, S, and G2/M phases were determined by flow cytometry.

### Transwell migration and invasion assays

Before assessing cell invasive ability, transwell chambers (Corning Incorporated, Corning, NY, USA) were coated with 50 μL Matrigel (354480; BD Biosciences) and incubated at 37°C for 1 h. Next, 5 × 10^4^ cells resuspended in 200 μL FBS-free culture medium were seeded in the upper chamber. The bottom chamber was filled with 500 μL culture medium containing 20% FBS as a chemoattractant. After incubating the chambers for 24 h, noninvasive cells in the upper chamber were eliminated with a cotton swab. Invasive cells were fixed in 4% paraformaldehyde, stained with 0.5% crystal violet, and imaged under an inverted microscope. The, invasive cells in five randomly selected fields were counted. Transwell migration assay was performed in the same manner as transwell invasion assay, except that the chambers were not precoated with Matrigel.

The article "LINC00514 drives osteosarcoma progression through sponging microRNA-708 and consequently increases URGCP expression" was retracted in 2024. Reasons: plagiarized images; overlap with other authors' work; signs of a paper mill; concerns about the images.

### Tumor xenograft model

Lentiviral vectors encoding a sh-LINC00514 or sh-NC were packaged by GeneChem Co., Ltd. HOS cells were transfected with lentiviral vectors carrying sh-LINC00514 or sh-NC. Cells with stable LINC00514 knockdown were selected with puromycin.

Four-week-old male BALB/c nude mice (Shanghai Lingchang Biotech Co., Ltd.; Shanghai, China) were subcutaneously injected with HOS cells stably expressing sh-LINC00514 or sh-NC. Each group contained three nude mice. The mice were raised under specific pathogen-free conditions. The width and length of subcutaneous tumor xenografts were measured every 4 days starting from day 7 after inoculation. Tumor volume was calculated using these measurements with the following formula: tumor volume = 0.5 × width^2^ × length. One month after inoculation, all mice were euthanized and the tumor xenografts were excised and weighed. The total RNA and protein was extracted from tumor xenografts (one month after cell injection) and genes expression status was monitored.

### Bioinformatics prediction

StarBase version 3.0 (http://starbase.sysu.edu.cn/) was used to analyze LINC00514–miRNA interactions.

### Luciferase reporter assay

LINC00514 fragments harboring the WT and mutant miR-708-binding sites were designed and chemically synthesized by Shanghai GenePharma Co., Ltd. The WT and MUT LINC00514 fragments were cloned into the pmirGLO Dual-luciferase Target Vector (Promega Corporation, Madison, WI, USA) to produce WT-LINC00514 and MUT-LINC00514 reporter plasmids, respectively. After culture in 24-well plates, WT-LINC00514 or MUT-LINC006514 was cotransfected into cells with miR-708 mimic or miR-NC using Lipofectamine® 2000. At 48 h after transfection, luciferase activity was assayed using the Dual-Luciferase Reporter Assay System (Promega Corporation). *Renilla* luciferase activity was normalized to firefly luciferase activity.

### RIP assay

The binding interaction between LINC00514 and miR-708 in OS cells was assessed by the RIP assay using the Magna RIP™ RNA-Binding Protein Immunoprecipitation Kit (Millipore; Bedford, MA, USA). OS cells were lysed with complete RIP lysis buffer, and the lysates (100 μL) were incubated with magnetic beads labeled with a human anti-AGO2 or normal IgG antibody (Millipore). After incubation overnight at 4°C, the magnetic beads were rinsed with a wash buffer. The immunoprecipitate complex was treated with proteinase K buffer at 55°C for 30 min. The isolated coprecipitated RNA was analyzed using RT-qPCR to detect LINC00514 and miR-708.

### Western blotting

Total proteins were isolated using RIPA buffer supplemented with phenylmethylsulphonyl fluoride (both from Beyotime Institute of Biotechnology; Shanghai, China). Protein concentration was measured using a bicinchoninic acid assay kit (Pierce; thermo Fisher Scientific, Inc.). Proteins were separated by 10% SDS–PAGE and transferred onto polyvinylidene fluoride membranes. The membranes were blocked with 5% nonfat milk powder diluted in TBST at room temperature for 2 h. After washing thrice with TBST, the membranes were incubated with anti-URGCP (sc-376934; dilution 1:1000; Santa Cruz Biotechnology, Santa Cruz, CA, USA) and anti-GAPDH (sc-47724; dilution 1:1000; Santa Cruz Biotechnology) primary antibodies overnight at 4°C. Then, the membranes were incubated with a horseradish peroxidase-conjugated goat anti-mouse IgG secondary antibody (sc-516102; dilution 1:5000; Santa Cruz Biotechnology) at room temperature for 2 h. The Immobilon Western Chemiluminescent Horseradish Peroxidase Substrate (Millipore) was added to the membranes to visualize the blots. Quantity One software version 4.62 (Bio Rad Laboratories, Inc., Hercules, CA, USA) was utilized to analyze the protein signals.

The article "LINC00514 drives osteosarcoma progression through sponging microRNA-708 and consequently increases URGCP expression" was retracted in 2024. Reasons: plagiarized images; overlap with other authors' work; signs of a paper mill; concerns about the images.

### Statistical analysis

All assays were repeated at least three times. All results are presented as mean and standard deviation. Comparisons between 2 groups were conducted using Student’s *t*-test and those among ≥3 groups using one-way analysis of variance followed by Tukey’s post hoc test. Overall survival was analyzed using the Kaplan–Meier method, and differences between the curves were analyzed using the log-rank test. Correlations of LINC00514 expression with clinicopathological characteristics of OS patients were evaluated using the χ^2^ test. Spearman’s correlation analysis was performed to determine the correlation between LINC00514 and miR-708 expressions in OS tissues. *P*-value of <0.05 was considered statistically significant.

### Ethics statement

Our study was approved by the Institutional Research Ethics Committee of Shandong Provincial ENT Hospital. Written informed consent was provided by all patients or their families. All animal experiments were approved by the Animal Research Committee of Shandong Provincial ENT Hospital.
